# Novel Insights into the Molecular Features and Regulatory Mechanisms of Mitochondrial Dynamic Disorder in the Pathogenesis of Cardiovascular Disease

This article has been retracted.

**DOI:** 10.1155/2021/6669075

**Published:** 2021-02-20

**Authors:** Ying Tan, Fengfan Xia, Lulan Li, Xiaojie Peng, Wenqian Liu, Yaoyuan Zhang, Haihong Fang, Zhenhua Zeng, Zhongqing Chen

**Affiliations:** ^1^Department of Critical Care Medicine, Nanfang Hospital, Southern Medical University, Guangzhou 510515, China; ^2^Department of Cardiology, Shunde Hospital, Southern Medical University (The First People's Hospital of Shunde Foshan), Foshan, 528300 Guangdong, China; ^3^Department of Critical Care Medicine, Huiqiao Medical Center, Nanfang Hospital, Southern Medical University, Guangzhou 510515, China; ^4^Department of Anesthesiology, Nanfang Hospital, Southern Medical University, 1838 Guangzhou Ave N, Guangzhou 510515, China

## Abstract

Mitochondria maintain mitochondrial homeostasis through continuous fusion and fission, that is, mitochondrial dynamics, which is precisely mediated by mitochondrial fission and fusion proteins, including dynamin-related protein 1 (Drp1), mitofusin 1 and 2 (Mfn1/2), and optic atrophy 1 (OPA1). When the mitochondrial fission and fusion of cardiomyocytes are out of balance, they will cause their own morphology and function disorders, which damage the structure and function of the heart, are involved in the occurrence and progression of cardiovascular disease such as ischemia-reperfusion injury (IRI), septic cardiomyopathy, and diabetic cardiomyopathy. In this paper, we focus on the latest findings regarding the molecular features and regulatory mechanisms of mitochondrial dynamic disorder in cardiovascular pathologies. Finally, we will address how these findings can be applied to improve the treatment of cardiovascular disease.

## 1. Introduction

Mitochondria are highly dynamic organelles that not only by keeping adenosine triphosphate (ATP) levels but also by generating low levels of reactive oxygen species (ROS) for cell signaling and that dysfunction in either of these processes could lead to pathology [1, 2]. In 1914, Lewis M. and Lewis W. [3] first proposed the concept of mitochondrial dynamics, that is, the dynamic change process in which mitochondria constantly divide and fuse in the cell, thus, maintaining its stable morphology and network structure. In recent years, it has been reported that [3–5] factors that maintain cell homeostasis, in addition to mitochondrial fission and fusion, mitochondrial-endoplasmic reticulum structure coupling, mitochondrial biosynthesis, and mitophagy, are all related to mitochondrial morphology and cell homeostasis. Some scholars [4] included it in the concept of mitochondrial dynamics, while others [5] summarized all the above factors as mitochondrial dynamic-related functions. This review favors the latter, namely, the mitochondrial dynamics for the dynamic process of mitochondrial fission-fusion. Mitochondria are often arranged in parallel in the myocardium along the long axis of the cell, and their size is described by the length/width ratio of the mitochondria. The length/width ratio of fibroblast mitochondria was about 6, and the mitochondria of mature cardiomyocytes were oval (length/width value was about 1.5), smaller, and rounder than the mitochondria of fibroblasts [6]. In the body, mitochondrial structure is continuously reshaped through fission and fusion. Mitochondrial fusion will produce enlarged mitochondria (longer and larger), and the fission will produce shorter and smaller offspring mitochondria, which are called fragmented mitochondria [7]. Studies [8, 9] have shown that mitochondrial dynamics is involved in mitochondrial maintenance, biological productivity, and cell death. The dynamic balance of mitochondria maintains the homeostasis of cardiomyocytes. Once it is out of balance, which will have a great impact on the pathogenesis of cardiovascular diseases. Moreover, mitochondria are not only the main energy-producing organelles in cells but also critical regulators of cardiomyocytes in response to various stimuli such as hypoxia, oxidative stress, and hyperglycemia [10]. The latest research showed that the imbalance of mitochondrial dynamics is closely associated with the occurrence and development of various cardiovascular diseases, including ischemia-reperfusion injury, atherosclerosis, diabetic cardiomyopathy, septic cardiomyopathy, hypertrophic cardiomyopathy, and heart failure [4] (Figure 1).

## 2. Mitochondrial Fusion and Fission Machinery

The processes of mitochondrial fusion and fission are highly controlled by the molecular machinery. It was found that the proteins related to mitochondrial dynamics are all important members with the function of Guanosine triphosphatases (GTPase), including (1) mitofusin 1 (Mfn1) and mitofusin 2 (Mfn2) are the proteins that regulate the fusion of mitochondrial outer membrane, which are located in the mitochondrial outer membrane and formed three different molecular compounds, namely, Mfn1 oligomers, Mfn2 oligomers, and Mfn1-Mfn2 oligomers; these compounds can promote mitochondrial fusion process [11]. The Mfn1 and Mfn2 proteins have an N-terminal GTPase domain, and the C-terminal part induces mitochondrial fusion protein oligomerization. Mfn2 is also associated with myocardial cell apoptosis and mitochondrial autophagy. (2) Optic atrophy 1 (OPA1) is the protein that regulates the fusion of mitochondrial intima, which can not only ensure the stability of mitochondrial intima structure but also participate in the remodeling of mitochondrial cristae. OPA1 mainly exists in two forms: long OPA1 (long OPA1 protein structure, L-OPA1) and short OPA1 (short OPA1 protein structure, S-OPA1). Under the action of intestinal peptidase OMA1 and I-AAA proteolytic enzyme YME1L, L-OPA1 can be hydrolyzed into S-OPA1. The former is anchored on the mitochondrial inner membrane to regulate intimal fusion, while the latter is located in the membrane space, promoting mitochondrial fragmentation and fission [12]. (3) The protein regulating mitochondrial fission is Drp1, a member of the GTPase family, which is located in the cytoplasm and participates in the fission of the mitochondrial outer membrane. It is produced by DNM1L gene coding. Drp1 mainly contains four regions from the N-terminal to the C-terminal: GTPase region, intermediate region, polytropic region, and GTPase effector region. Unlike Mfn, Drp1 lacks a lipid-interacting hydrophobic transmembrane domain and must bind to other receptor proteins to be recruited into the mitochondrial outer membrane [13]. Studies [14] showed that Drp1 had dimer or tetramer under basic conditions and further self-assembled in the fission process to form a larger poly structure. The latter promoted outer membrane fusion and separation through GTP, depending on conformational changes. Mitochondria repair damaged mitochondria through mutual fusion, and self-fission is conducive to the removal of irreparably damaged mitochondria. However, mitochondrial fission first fragments the irreparable mitochondria and then removes the fragmented mitochondria from the cell to maintain the quality of the mitochondria, thereby protecting the normal function of the mitochondrial network [15].

In mammalian cells, mitochondrial fission is regulated by Drp1 and mitochondrial fission 1 protein (Fis1), mitochondrial fission factor (Mff), and mitochondrial dynamic proteins 49 and 51 (MiD49/51) [16]. In the early stage of mitochondrial fission, Drp1 acts as a mechanical enzyme similar to dynein, which plays a role in constricting the mitochondrion physically. Because Drp1 lacks a mitochondrial target sequence, it needs to form a fission complex with Fis1 located on the outer mitochondrial membrane [17]. However, studies in mammalian cells have found that silencing Fis1 has little effect on Drp1 transport to mitochondria [18]. At this point, Mff seems to be a mitochondrial receptor protein for Drp1 [19]. Decreased MFF levels induce mitochondrial elongation and reduce Drp1 transport to mitochondria [19]. Similarly, MiD49 and MiD51 are also involved in the fission mechanism in mammals [20] (Figure 2). At present, it has been widely recognized that multiple receptors can recruit Drp1 to mitochondria to induce mitochondrial fission. Posttranslational modifications can also modify the activity of Drp1. Cdk1/cyclin B kinase [21] and CaMKI*α* [22] increase Drp1 mitotic activity. On the contrary, phosphorylation of cyclic AMP-dependent protein kinase (PKA) reduces the function of Drp1 [23]. Specifically, Ca^2+^-calmodulin-dependent phosphatase calcineurin can remove this phosphate residue and promote mitochondrion fission [24].

## 3. Effects of Mitochondrial Dynamic Imbalance on the Organism

Numerous studies [25] have shown that mitochondrial fusion is beneficial to oxidative phosphorylation. Mitochondrial fusion can prevent mitochondrial DNA loss and protect mitochondrial protein synthesis and thus maintaining normal mitochondrial function. Besides, the mitochondrial fusion event can dilute the damaged mitochondrial proteins and DNA and repair the damaged mitochondria through the process of “functional complementation” [9]. Damage to the mitochondrial fusion mechanism can accelerate mitochondrial fission and then produce mitochondrial fragmentation leading to the loss of oxidative phosphorylation and apoptosis of cardiomyocytes. A study [26] found that inducing Drp1 gene mutation in mice can affect mitochondrial function and induce mitochondrial autophagy, leading to cardiac dilatation and heart failure. Inhibiting Drp1-induced mitochondrial fission with Drp1 inhibitor (Mdivi-1) or other drugs has a protective effect on injured heart and brain after ischemia [27, 28]. At this point, the mitochondrial fission seems to be “harmful.” However, many studies [29, 30] have reported that knockout of myocardial Drpl gene can cause fission disorder, which produces large, long, and dysfunctional mitochondria, and finally leads to heart failure and death. It is obvious that the mitochondrial fission is equally important for the maintenance of cardiac function.

Excessive mitochondrial fragmentation is involved in most heart diseases, thus, enhancing mitochondrial fusion will be a potential therapeutic strategy. The latest research found mitochondrial fusion provoked by fusion promotion and fission inhibition direct the different fate of heart, Mfn2 upregulation other than Drp1 downregulation well maintains heart mitochondrial function is a more safe strategy for correcting excessive mitochondrial fragmentation in hearts [31]. Maneechote's team intervened rats with ischemia-reperfusion using mitochondrial fusion promoter M1 (2 mg/kg). They found that the administration of M1 before ischemia reduced the infarct size and cardiac apoptosis and exerted the greatest cardioprotective effect. This indicates that myocardial ischemia-reperfusion injury can be reduced by increasing mitochondrial fusion [32]. However, excessive mitochondrial fusion can also lead to disease. Studies have shown that the point mutation of L341P could promote the rapid degradation of SLC25A46. As a mitochondrial carrier protein, the decreased expression of SLC25A46 may promote the stability and oligomerization of Mfn1 and Mfn2 on mitochondria, thereby leading to excessive mitochondrial fusion and ultimately manifested as a rare disease of cerebellopontine hypoplasia [33]. In addition, increased mitochondrial fusion can lead to increased oxidative stress and abnormal Ca^2+^ homeostasis [34, 35], which can lead to arrhythmias, especially atrial fibrillation [36, 37]. Therefore, the effect of mitochondrial dynamics on the myocardium depends on the proper balance between mitochondrial fusion and fission which cannot be divided. In this process, mitophagy also plays a key role, which can remove the fragmented mitochondria caused by mitochondrial fission. Once the mitochondrial autophagy is impaired or the mitochondria divide excessively, the excessive accumulation of the fragmented mitochondria will cause heart damage.

Mitophagy is the selective sequestration of mitochondria by autophagosomes and is degraded by lysosomes to remove damaged mitochondria [38, 39]. Excessive mitochondrial fission causes increased mitochondrial debris, resulting in abnormal energy metabolism and apoptotic events. In contrast, mitophagy can remove injured mitochondrial fragmentation and thus render the IR-damaged microvasculature less sensitive [40]. A study showed nuclear receptor subfamily 4 group A member 1 (NR4A1) could promote Drp1 activation and inhibit BCL2 interacting protein 3 (Bnip3) transcription, resulting in excessive Drp1-associated fission and defective Bnip3-depended mitophagy [41]. Currently, there are two main opinions on the relationship between mitophagy and mitochondrial fission: “fission-regulated autophagy,” that is, mitochondria form small fragments through fission, so that mitophagy can more easily clear the mitochondrial fragments; “autophagy resists fission,” mitochondria are fragmented after fission, and the fragmented mitochondria contain incomplete mitochondrial DNA genes and damaged mitochondrial membrane potential. These have become the main removal target of mitophagy [42, 43]. However, the current research results cannot fully explain whether mitochondrial autophagy can remove the mitochondrial debris, thereby preventing cardiovascular damage.

## 4. Mitochondrial Dynamics and Cardiovascular Disease

### 4.1. Myocardial Ischemia-Reperfusion Injury(IRI)

Most clinical studies using ischemia regulation and related drugs to reduce infarct size have not been successful; therefore, coronary artery microvascular damage as a target of auxiliary cardiac protection has become the focus of attention [44]. During ischemia, myocardial cells are dominated by anaerobic glycolysis, leading to the accumulation of acid products, the depletion of adenosine triphosphate (ATP), calcium overload in the mitochondrial matrix, and the excessive production of ROS. Studies [45] showed that ROS and calcium overload may regulate mitochondrial dynamic changes by mediating the expression of mitochondrial dynamic-related proteins, thus, playing an important role in myocardial ischemia-reperfusion injury. Mitochondrial fission may cause abnormal mitochondrial energy metabolism, promote apoptosis of myocardial cells, and lead to ventricular remodeling after myocardial infarction. Wang et al. confirmed that the regulation of miR-499 level can affect the degree of apoptosis and myocardial infarction and cardiac dysfunction caused by ischemia-reperfusion (I/R) according to targeting calcineurin-mediated Drp1 activation [46]. It has been found that [47] the level of Drpl protein in the cytoplasm of mouse cardiomyocytes and its phosphorylated protein levels were decreased, while the level of Drp1 protein in the mitochondrial outer membrane was increased, which indicates that the level of miR-499 can affect the degree of apoptosis and myocardial infarction. The decrease in its expression causes the activation of calcineurin, promotes the dephosphorylation of Drp1, and produces fragmented mitochondria. In addition, using mdivi-1 to inhibit Drp1 can increase the proportion of extended mitochondria in cardiomyocytes, delay the opening of mitochondrial permeability transition pore (mPTP), reduce acute IRI-induced cell death, and reduce the area of myocardial infarction caused by IRI, indicating that the inhibition of Drp1 has potential therapeutic effect.

In the reperfused heart, calcium overload is an effective regulator of Drp1 after reperfusion. In the cytoplasm, the accumulation of Ca^2+^ activates calcineurin and dephosphorylates Drp1 (S637), leading to mitochondrial fission and cell apoptosis. mir-499 can offset the effect of calcium overload on Drp1 activity, but the expression of mir-499 is reduced and is more sensitive to IRI [46]. To keep mitochondrial integrity and prevent cardiomyocytes from apoptosis, activation of PIM-1 is used to inhibit Drp1 and prevent mitochondrial fission. In response to IRI, calcium overload mainly targets Drp1, while ROS mainly targets Mfn and OPA1. Mfn1 and Mfn2 are necessary for mitochondrial fusion, but they have opposite effects in IRI, possibly due to the fission effect of Mfn2. Mfn2 upregulates ROS during IRI, which is sufficient to induce cardiomyocyte apoptosis by inhibiting Akt and activating caspase-9. Mfn2 knockout delays mitochondrial membrane permeability and the opening of mPTP to prevent myocardial cells from being affected by IRI. ROS upregulates the level of miR-140, downregulates the Mfn1 expression in the IR heart, disconnects the mitochondrial network, and intensifies myocardial cell apoptosis. ROS activates OMA1, while L-OPA1 is completely sheared into a short soluble S-OPA1, leading to remodeling of mitochondrial cristae and release of cytoplasmic C. There are three Bcl-2 family proteins, namely, Bnip3, Bak, and Bax, which lead to mitochondrial dynamic imbalance and mitochondrial cristal remodeling and further promote mitochondrial dysfunction and cardiomyocytes death, all of which are associated with IRI [48]. In the process of IRI, Mfn2 increases with the rise of ROS. Induction of myocardial apoptosis by inhibiting Akt and activating Caspase-9, as well as increasing Mfn2 levels, is necessary and sufficient.

It has been reported that the level of OPA1 in heart samples from patients with ischemic cardiomyopathy is decreased [49]. However, according to the contradictory and unexpected findings, the role of mitochondrial fusion proteins (Mfn1, Mfn2, and OPA1) as cardiac protective targets is still controversial. In HL-1 cells, the overexpression of Mfn1 or Mfn2 delays the opening of mPTP and reduces I/R-induced cardiomyocyte death [50]. However, in a parallel study, Papanicolaou et al. reported that small interfering RNA (siRNA) knockout of Mfn2 prevented mPTP opening, thereby making cardiomyocytes more vulnerable to ROS [51]. Similarly, some studies have reported that partial gene ablation of Opa1 can prevent mPTP opening; however, the effect on acute ischemic reperfusion has not been explored [52]. In short, the interaction between mitochondrial fusion proteins and I/R is complicated, which needs further study.

### 4.2. Cardiac Hypertrophy and Failure

Cardiac hypertrophy is caused by multiple stimuli such as hemodynamic overload, ischemia, and activation of neurohormones. Cardiac hypertrophy was initially considered adaptive, and it involved these changes in the structure, morphology, and function of cardiomyocytes, which ultimately led to an increase in heart mass [53–55]. Initially, as a compensatory process, hypertrophic growth normalizes oxygen demand and wall stress. But long-term exposure to disease-related stimuli ultimately leads to pathological cardiomyocyte growth and heart failure [56].

In cardiomyocytes of adults, mitochondria are tightly packed between myofibrils [57], and it was reported that no mitochondrial dynamic events occurred in this subpopulation of mitochondria [58]. However, significant changes in mitochondrial dynamics can be found in models of cardiac hypertrophy [54] and heart failure. Chen et al. [49] found fragmented mitochondria associated with reduced OPA1 levels in both rat and human models of heart failure. In other studies of neonatal rat cardiomyocytes exposed to phenylephrine to induce cardiomyocyte hypertrophy and in vivo models of cardiac hypertrophy, it was also found that the level of Mfn2 mRNA decreased [59]. A recent study found miR-485-5p regulates mitochondrial fission in a mice model of cardiac hypertrophy induced by phenylephrine through targeting mitochondrial anchored protein ligase [60].

Calcineurin is an important regulator of cardiac hypertrophy and heart failure, and it involves in the regulation of mitochondrial fission through Drp1 dephosphorylation. Wang et al. reported that the A and B subtypes of the calcineurin catalytic subunit are both direct targets of miR-499, promoting the phosphorylation of Drp1 at residue Ser 656, thus inhibiting mitochondrial fission [46]. Interestingly, the miR-499 transgenic mice showed decreased hypertrophy parameters after ischemia-reperfusion (I/R). Conversely, knocking out endogenous miR-499 can intensify maladaptive cardiac remodeling [46]. Recently, a study showed that noradrenaline induces mitochondrial fission by calcineurin-and Drp1-dependent manner. Adenovirus-regulated dominant-negative Drp1 expression inhibits norepinephrine-induced mitochondrial fission and hypertrophic cardiomyocyte growth. In addition, adenoviruses expressing antisense sequences of Mfn2 are enough to promote mitochondrial fission and cause hypertrophic responses in cultured myocardial cells [61]. Consistent with these findings, Papanicolaou et al. confirmed that moderate myocardial hypertrophy with mild functional deterioration appears in Mfn2 knockout mice [51]. In a recent study, heart failure was induced by ascending aorta cerclage in wild-type mice, followed by treatment using Drp1 inhibitor mdivi-1, which showed that mdivi-1 treatment alleviated left ventricular dysfunction, and these effects were considered to be associated with reduced expression of the autophagy markers LC3 and p62 [62]. These findings reported in this review indicate the major role of mitochondrial fission in pathological cardiac remodeling. In addition, a recent study showed that microRNA-20b intensified cardiac hypertrophy by downregulating Mfn2 and promoting cytoplasmic Ca^2+^ overloading, weakening mitochondrial buffering capacity [63].

Heart failure (HF) is the terminal stage of various cardiovascular diseases, characterized by high morbidity, mortality, and rehospitalization rate. The currently recognized as the pathogenesis of heart failure includes overactivated nervous and humoral system, immune regulation disorder, energy metabolism disorder, oxidative stress damage, among which both energy metabolism and oxidative stress damage mechanisms play a role in mitochondria. According to the analysis of heart tissues of patients with heart failure by electron microscopy, different degrees of mitochondrial damage such as the increased mitochondrial number and decreased volume were found, proving that the normal function of mitochondrial dynamic proteins (MDPs) plays an important role in mitophagy and metabolic regulation, and MDP deficiency can lead to dilated cardiomyopathy and heart failure.

If mitophagy is insufficient, cell homeostasis will be impaired, causing cardiomyopathy and HF. Mfn2 is an important mediator of mitophagy. It regulates mitophagy through the PINK1-Mfn2-Parkin signaling pathway, which plays a significant role in mitochondrial quality control and maturation [7]. Mitochondrial maturation is realized through the elimination of fetal mitochondria after birth. Mfn2-Parkin interaction promotes the widespread elimination of fetal mitochondria in the first 3 weeks after birth, which is considered as a prerequisite for the introduction of mature myocardial mitochondria needed for fatty acid metabolism. Mitochondrial quality control dependent on Mfn2 is achieved by eliminating stress-induced mitochondria, leaving healthy mitochondria to refuse. In addition to Mfn2, Drp1 for mitophagy induction is also essential; this can control the quality of mitochondria and prevent heart failure. Drp1-induced mitochondrial fission can produce a group of tiny mitochondria which can be separated by autophagosomes and then be degraded by lysosomes. It can be seen that mitochondrial fission induced by Drp1 is a prerequisite for mitophagy [64]. Mitophagy was further validated in the TAC model; among them, the deficiency of Drp1 resulted in mitophagy dysfunction and exacerbated the progress of mitochondrial and cardiac dysfunction.

Cardiomyocytes mainly rely on fatty acid metabolism to keep their normal function, and increased glucose utilization is harmful to heart function, resulting in dilated cardiomyopathy [65]. MDPs have been identified as a major regulator of cardiac metabolic state, and active mitochondria may be caused by MDP-mediated metabolic regulation. Compared with adult cardiomyocytes, neonatal cardiomyocyte metabolism requires more glucose to promote heartbeat. During the development of the postpartum heart, it is mainly the conversion of sugar decomposition to fatty acid metabolism. PINK1-Mfn2-Parkin-dependent autophagy helps adult mitochondria replace fetal mitochondria and promote the transformation of metabolism. The latter provides enough energy to the adult heart for maintaining the normal function; otherwise, it will lead to dilated cardiomyopathy. The end stage of heart failure is characterized by the transition from fatty acid metabolism to glucose metabolism. A recent study [66] found OPA1 dysfunction leads to metabolic abnormality. Specific ablation of YME1L in the mouse heart can activate OMA1, promote the hydrolysis of OPA1 protein, and further induce mitochondrial fragmentation, thus, determining the tendency of the mitochondrial substrate to cell energy demand (fatty acid to glucose). Changes in mitochondrial metabolism and cardiac function can be saved by loss of OMA1, which is promoted by lowering the OPA1 cleavage. The balance of OMA1 and YME1L content is essential for OPA1 to regulate mitochondrial fusion. The specific knockout of the YME1L gene in myocardial tissue can enhance the activity of OMA1, eventually leading to dilated cardiomyopathy and heart failure.

### 4.3. Diabetic Cardiomyopathy

Mitochondrial fission occurs in diabetic cardiomyopathy, and negative regulation of mitochondrial fusion protein may be caused by reduced PGC-1 expression in diabetic cardiomyopathy. In diabetic cardiomyopathy, decreased OPA1 protein level was detected even though the protein Drp1 and/or Fis1 did not follow this reduced expression pattern [67]. Mitochondria fusion promoter M1 can effectively restore mitochondrial dynamic balance and ameliorate diabetic cardiomyopathy in an Opa1-dependent way [68]. Impaired insulin signaling, such as insufficient insulin production (type 1 diabetes mellitus, T1DM) and/or insulin resistance (type 2 diabetes mellitus, T2DM), can lead to elevated blood sugar levels, often referred to as hyperglycemia. Insulin signaling maintains a normal mitochondrial network, while hyperglycemia leads to mitochondrial fission. Insulin regulates heart metabolism by stimulating glucose uptake and directly regulating mitochondrial function. Insulin treatment improves OPA1 protein level, promotes mitochondrial fusion, increases *ΔΨ*m, and raises the level of ATP and oxygen consumption of cardiomyocytes in vivo. Insulin activates the Akt-mTOR-NF*κ*B-OPA1 signaling pathway, leading to mitochondrial fusion and promoting mitochondrial oxidation. Silent OPA1 prevents the insulin-induced all metabolic effects, which phosphorylates Drp1 by activating MAP kinase ERK1/2 and ROCK1 under persistent hyper glucose conditions, leading to mitochondrial fission, ROS production, and cell death. Also, NRCMs grown in medium with high glucose concentration showed low protein levels of OPA1 and more fragmented mitochondria [65], which is similar to the mitochondrial changes observed in heart biopsies of patients with type 2 diabetes.

In contrast, activation and/or elevated Drp1 expression leads to insulin resistance. In addition, the hereditary and pharmacological inhibitory effects of skeletal muscle cells attenuate Drp1-induced mitochondrial fission, membrane potential depolarization, and insulin resistance [69]. Drp1 induces mitochondrial dysfunction and myocardial insulin resistance to mediate mitochondrial fission. Besides, Mfn2 deficiency further leads to insulin resistance, promotes mitochondrial dysfunction, increases H_2_O_2_ level, and activates JNK, which leads to insulin resistance in skeletal muscles. Exercise can inhibit mitochondrial fission protein levels and prevent phosphorylation of Drp1 at S616 [70], thus, improving fat oxidation and insulin sensitivity in the heart. The specific role of mitochondrial fission in insulin resistance in the body needs further research.

Mitochondrial dynamics has a direct impact on pancreatic function. In ob/ob mice, the level of OPA1 in islet cells decreased before the onset of diabetes [71]. Silencing the OPA1 gene in islet beta cells could generate similar results [72]. OPA1 deficiency in beta cells maintained normal mtDNA copy numbers; however, there has a significant decrease in complex IV activity and levels of electron transport chain, resulting in reduced insulin secretion and ATP production. Whether mitochondrial fission contributes to diabetic cardiomyopathy-related cardiac dysfunction remains unclear. Similarly, whether mitochondrial fusion acts as a direct mediator of mitochondrial metabolism and heart function remains unclear. However, recent reports indicate that mitochondrial fragments are the “starting point” of many events involved in cardiometabolic diseases [67]. Increased fragmented mitochondria and reduced mitochondrial fusion proteins were observed in atrial tissue from patients with T2DM [73]. In a mouse model of cardiac lipotoxicity, correspondingly, more mitochondrial fragmentation were found, which was attributed to increased mitochondrial fission and decreased fusion [74]. In the early stages of insulin resistance, systolic dysfunction is observed in patients with type 2 diabetes but not in obese patients with metabolic healthy [67]. Thus, it is speculated that the decline in ventricular function during the transition from obesity to diabetes is at least partly caused by the deterioration of cardiomyocyte mitochondrial function. Further researches are needed to prove whether adjustment of mitochondrial dynamics may emerge as an intervention to improve mitochondrial performance and cardiac function.

### 4.4. Atherosclerosis

Atherosclerosis, a chronic inflammatory disease, is a key risk factor for early death [75]. In this complicated disorder, increased levels of adhesion molecules in arterial endothelium were expressed, promoting the infiltration, differentiation, and transformation of monocytes into highly active lipid foam cells, accompanied by VSMC migration to the intima [75]. Mitochondrial ROS production is a necessary factor for mitochondria to play a role in vascular diseases [76, 77]. In contrast, mitochondrial DNA is likely the most sensitive target of ROS [78, 79]. A recent study suggests that impaired mitochondrial DNA can directly exacerbate atherosclerosis. Ballinger et al. reported that impaired mitochondrial DNA was associated with the degree of atherosclerosis in both mouse models of early atherosclerosis and human aortic specimens [80]. In mice lacking apolipoprotein E, increased mitochondrial DNA damage and intensified atherosclerosis are associated with the deficiency of mitochondrial antioxidant enzyme manganese SOD [80]. Elevated mitochondrial ROS level also leads to endothelial cell dysfunction, accompanied by the proliferation and apoptosis of macrophages and VSMCs, which in turn result in the progression of atherosclerotic lesions and may cause plaque rupture [81]. In direct connection with this, Shenouda et al. observed increased mitochondrial fragmentation and Fis1 protein levels in venous endothelial cells of T2DM patients, and elevated abundance of Drp1 and Fis1 protein in human aortic endothelial cells pretreated with high glucose [82]. The changes in mitochondrial dynamics are associated with the increase in mtROS production. Silencing the expression of Fis1 or Drp1 with siRNA can prevent alterations in ROS production and mitochondrial network induced by high glucose [82]. Overall, these findings suggest mitochondrial fission plays a significant role in the pathogenesis of vascular diseases.

### 4.5. Septic Cardiomyopathy

Sepsis refers to systemic inflammatory response syndrome caused by a bacterial infection, and severe sepsis can lead to multiple organ failure [83]. Myocardial damage secondary to sepsis is called septic cardiomyopathy or sepsis-induced myocardial dysfunction [84]. Studies [85] reported that the mortality increased significantly during septic cardiomyopathy. In sepsis, the first manifestation of myocardial mitochondria is increased mitochondrial fission and fragmentation. Oxynitride (peroxynitrite, ONOO^−^) is produced along with the increase of oxynitride during sepsis. Continuous high levels of ROS and reactive nitrogen species (RNS) in mitochondria can directly damage mitochondrial components, including permanent inactivation of mitochondrial semifinished protein and mitochondrial membrane structure damage of mitochondrial DNA (mtDNA) and lipid bimolecular [86], resulting in inhibited function of the mitochondrial respiratory chain and decrease of mtDNA replication number, accelerating the generation of free radicals, which lead to the formation of a vicious cycle of free radical generation, mitochondrial structure destruction, and free radical generation. Studies [87] found that oxidative stress and nitriding stress can lead to increased mitochondrial division and fragmentation. In the early stage, when the body suffers stress factors, the first adaptive change of mitochondrial fission and fusion is triggered, that is, functional compensation is carried out through fusion. When the mitochondrial damage is excessive, mitochondrial fission increases, inducing mitochondrial fragmentation and initiating autophagy mechanism for recycling. Mitochondrial fission is far greater than fusion when mitochondrial injury is excessive, followed by a large number of fragmented mitochondria accumulate in cells and cannot be removed. The activation of cell apoptosis and necrosis signal lead to irreversible damage of the body [88].

Secondly, the influence of sepsis on mitochondrial dynamics is also manifested in the abnormal expression of mitochondrial dynamic regulatory proteins. Studies [89, 90] reported that lipopolysaccharide (LPS) promoted mitochondrial fission in the model of lung injury induced by sepsis, leading to increased Drpl mRNA and protein expression, while Mfn1, Mfn2, and OPAl mRNA and protein expression were decreased. In the model of sepsis-induced myocardial injury, mitochondria underwent morphological changes in the early stage of the disease, which showed the destruction of mitochondrial double-membrane structure, matrix edema, and transparency. Then, mitochondrion fission and fusion were unbalanced, and a large number of fragmented mitochondria accumulated in cardiomyocytes. This change was related to the increase of phosphorylated Drpl expression, but not to Mfn2, there was no significant change in Mfn2 expression [91, 92]. Recent research observed that mitochondrial dynamics changed significantly with the progression of sepsis, and this change was parallel to the change of oxygen and nitrogen free radicals [88]. In the model of sepsis-induced liver injury, tubular mitochondria decreased by 45% and globular mitochondria (fragmented mitochondria) increased by 46% in the LPS group at 6 h (NO level reached the maximum). At the same time, the expression of Mfn2 mRNA decreased significantly, while the Drpl mRNA did not change significantly; the percentage of ball and rod-shaped mitochondria recovered in the LPS group at 24 h, with little difference, compared with the control group. At this time, Mfn2 mRNA expression increased compared with 6 h, and there was no difference with the control group [88]. In the cecal ligation and perforation group, the tubular mitochondria decreased by 65%, and the globular mitochondria increased by 100% at 12 h (the maximum value of NO). At this time, the expression of Mfn2 mRNA was significantly decreased while the Drpl mRNA was significantly increased. With the progression of the disease, mitochondrial morphology cannot be restored, the percentage of globular mitochondria was still increased, and the expressions of Mfn2 mRNA and Drp 1mRNA did not change much compared with 12 h [88]. This indicates that changes in mitochondrial dynamics may reflect the degree of progression of the disease to some extent.

At present, there is no specific treatment for sepsis-induced myocardial injury, and the current treatment can only relieve the symptoms of patients, but cannot fundamentally reverse the changes of cardiomyocytes at the molecular level. Studies [93] confirmed that cardiac function can be successfully restored in patients even if the myocardial structure has been changed. A new viewpoint [93] holds that the failing cardiomyocytes as “dysfunctional but alive” tissue, rather than being irreversibly damaged tissue. This perspective can help us break away from traditional therapeutic thinking and design therapies that target cardiomyocytes. Studies [50] showed that the inhibition of the Drpl gene and transfection of Mfn1and Mfn2 gene can prolong mitochondria of cardiomyocytes and delay the opening of mPTP, thereby reducing myocardial injury. Canfield and his team found Mdivi-1 reduced the area of myocardial infarction by using Mdivi-1 to regulate mitochondrial dynamics [94]. Chen and his team first proved that knockout of Mfn1 or Mfn2 reversed myocardial injury caused by homozygous mutation of the Mff gene [8]. These findings show that myocardial injury may be reversed if measures are taken before the mitochondrial dynamic imbalance reaches uncontrollably (cells are on the verge of death). The mechanisms of myocardial injury in sepsis are complex and include almost all aspects of the physiological changes of cardiomyocytes, among which mitochondrial dysfunction is the core. Mitochondrial dynamics are involved in the energy metabolism process of cardiomyocytes, and the imbalance of its fission and fusion will cause insufficiency of cell energy supply and then appear function dysfunction. Sepsis-induced myocardial injury is related to the imbalance of mitochondrial dynamics, and resetting its fission and fusion balance site is expected to be a new intervention target for the prevention and treatment of septic cardiomyopathy.

## 5. Concluding Remarks

Mitochondrial dynamics has a crucial effect on the homeostasis of the cardiovascular system, which is related to important cellular functions such as mitochondrial quality control and metabolism. The underlying molecular mechanisms of cardiovascular disease associated with mitochondrial dynamics may be quite different. For example, mitochondrial fission is triggered by the descending effect of hyperglycemia and insulin signaling pathway in diabetic cardiomyopathy; while in IRI, mitochondrial fission is mainly caused by Ca^2+^ overload and increased ROS production; while in HF, insufficient mitochondrial autophagy induced by Mfn2 and abnormal expression of OPA1 will lead to abnormal accumulation of mitochondrial fragment. Therefore, specific treatments for different MDP are necessary in order to improve mitochondrial dynamics and cardiac function. Mitochondrial fusion and fission proteins induce cardiomyopathy independent of mitochondrial dynamics under certain conditions. After treatment of oxidative stress, the increase of Mfn2 protein is associated with mitochondrial fission but not to mitochondrial fusion. Similarly, the OMA1-OPA1 signal causes dilated cardiomyopathy according to independent cell metabolism disorder with mitochondrial fission [67]. Thus, manipulating mitochondrial dynamics is not only a treatment strategy designed to optimize cardiovascular disease.

The mitochondrial fission has been observed in cardiovascular disease, but it is not clear whether restoring mitochondrial fusion alone could reverse cardiac pathogenesis. It is widely recognized that mitochondria undergo asymmetric fission, producing both normal mitochondria and dysfunctional mitochondria; among them, the impaired mitochondria are targeted for clearance through the Parkin/Pink protein complex [9]. Therefore, the mitochondrial fission is a prerequisite for Parkin/Pink mediated mitophagy, which is crucial for mitochondrial quality control in different cardiovascular diseases. Compared with mitochondrial fission, mitochondrial fusion has a certain beneficial effect, such as inhibiting the release of cytochrome C and improving mitochondrial metabolism, but mitochondrial fusion prevents the selective clearance of damaged mitochondria through mitophagy. It is widely believed that proper mitochondrial fission is protective for cardiomyocytes under stress, while excessive enhancement of fusion result in the accumulation of impaired mitochondria and accelerated progression of cardiomyopathy. It has been suggested that the combination therapy by reducing ROS production and maintaining proper mitochondrial fusion may improve the treatment of cardiovascular disease. Most data have confirmed that some chemical compounds have great potential for the regulation of mitochondrial dynamics. It has been confirmed that using the effective chemical compounds can treat some diseases in animal models [95], such as Mdivi-1, a small molecule inhibitor of Drp1, can relieve myocardial IRI in mice. Injection of Mdivi-1 into rats in advance can increase the length of mitochondria of cardiomyocytes in mice and reduce the area of myocardial infarction in ischemic mice by more than half [96]. Chemical compounds that inhibit OMA1 have therapeutic values on a variety of diseases, and effective OMA1 inhibitors protect normal mitochondrial networks and inhibit the release of cytochrome C by tightening mitochondrial cristae connections.

In brief, we focus on here evidence for new interventions targeting mitochondrial dynamics with relevance to some cardiovascular diseases. Furthermore, insights into mitochondrial dynamics will reveal new approaches to therapeutic manipulation of cardiomyocyte energetics, mitochondrial quality control, and function.

## Figures and Tables

**Figure 1:** Mitochondrial dynamics in cardiovascular disease. Mitochondria dynamic disorder is relevant to various aspects of cardiovascular biology, including cardiac development, responses to ischaemia/reperfusion (I/R) injury, cardiac hypertrophy and failure, type 2 diabetes mellitus (T2DM), atherosclerosis, and sepsis. In addition, mitochondrial fission is required for mitophagy.

**Figure 2:** The dynamic balance of mitochondrial fission and mitochondrial fusion maintains the proper function of complex organelle. Mitochondrial fusion is mainly regulated by mitofusin (Mfn) 1 and 2 and optical atrophy protein 1 (OPA1). Mitochondrial fission is mainly regulated by Drp1, Drp1, and its adapter proteins Fis1, Mff, and MiD49/51 control mitochondrial fission. This process is required by various cell processes, such as redistribution of mitochondria in mitosis and release of cytochrome c during cell apoptosis.
